This article has been retracted.

# Active Ingredient Paeonol of Jijiu Huiyang Decoction Alleviates Isoproterenol-Induced Chronic Heart Failure via the GSK3A/PPAR*α* Pathway

**DOI:** 10.1155/2023/3271057

**Published:** 2023-02-04

**Authors:** Wei Zhang, Manli Yu, Cenxi Zhang, Qing Yu, Sheng Xu, Qiongzhi Yan, Zhifu Guo, Yawei Xu

**Affiliations:** ^1^Department of Cardiology, Shanghai Tenth People's Hospital, Tongji University School of Medicine, China; ^2^Department of Cardiology, Changhai Hospital, Navy Medical University, China; ^3^Department of Cardiology, Second Affiliated Hospital of Naval Medical University, China; ^4^Department of Traditional Chinese Medicine, Shanghai Tenth People's Hospital, Tongji University School of Medicine, China

## Abstract

**Background:**

The pharmacological mechanism of the traditional Chinese medicine formula-Jijiu Huiyang decoction (JJHYD), which contains several herbal medicines for the treatment of chronic heart failure (CHF), is yet unknown. *Method and Materials*. The main active components of JJHYD were analyzed by ultrahigh-performance liquid chromatography-mass spectrometry (UHPLC-MS/MS). The target genes of JJHYD and CHF were retrieved through multiple databases, a drug-ingredient-target-disease network was created, and KEGG enrichment and GO analyses were carried out. The binding ability of paeonol and Glycogen Synthase Kinase-3 alpha (GSK3A) was confirmed by molecular docking. CHF animal model and cell model were constructed. The effects of paeonol on cardiac dysfunction, myocardial hypertrophy, cardiac lipid accumulation, and myocardial apoptosis were detected by echocardiography, histopathology, and flow cytometry, respectively. The effects of paeonol on the expression of myocardial hypertrophy index, GSK3A, and genes or proteins related to the PPAR*α* pathway were determined by qRT-PCR or western blot.

**Result:**

UHPLC-MS/MS analysis combined with database verification showed a total of 227 chemical components in JJHYD, among which paeonol was the one with heart-protective roles and had the highest content. Paeonol alleviated isoproterenol-induced cardiac lipid accumulation, cardiac hypertrophy, and myocardial dysfunction and inhibited the activation of the PPAR*α* pathway, while overexpression of GSK3A reversed these effects of paeonol. However, the reversal effects of GSK3A overexpression could be offset by siPPAR*α*.

**Conclusion:**

As the main active substance of JJHYD, paeonol participates in the protection of CHF by targeting the GSK3A/PPAR*α* signaling pathway to reduce lipid toxicity.

## 1. Introduction

Chronic heart failure (CHF) is a complex multifactorial clinical syndrome leading to abnormal heart structure and function, including left ventricular (LV) hypertrophy, the apoptosis of myocardial cells, and impaired ejection ability [1]. Myocardial metabolic abnormality is a key factor in the development of CHF, in which abnormal fat metabolism causes cardiac lipid accumulation, affecting cardiac contractile function and cardiac electrophysiological response [2]. At present, therapeutic drugs for CHF include diuretics, angiotensin-converting enzyme inhibitors, *β*-blockers, and digitalis drugs. [3]. Although the standardized treatment of CHF has improved the quality of life and prognosis of patients in recent years, novel strategies are still needed to be further explored to reduce the mortality and rehospitalization rate, as well as social and economic burdens.

Traditional Chinese medicine (TCM) exhibits several advantages in treating CHF since it has multiple targets, is inexpensive, and has less adverse reaction [4]. Jijiu Huiyang decoction (JJHYD) comes from *Yilingaicuo* (Correcting the Errors of Medicine) by Wang Qingren from the Qing Dynasty. JJHYD is composed of seven herbal medicines capable of reviving yang, supplementing qi, activating blood circulation, and resolving stasis. In addition to being used for treating shock caused by various reasons, it was shown to have good curative effects on heart failure (HF), myocardial infarction, and other heart diseases in clinics. However, it is currently unclear how JJHYD works to treat CHF from a pharmacological perspective.

Ultrahigh-performance liquid chromatography-mass spectrometry (UHPLC-MS/MS) combines the advantages of UHPLC (high resolution and fast analysis speed) and MS (strong qualitative ability and high sensitivity), providing an efficient and reliable method for component analysis, quality control, and pharmacokinetic studies of TCM [5, 6]. To thoroughly and systematically observe the intervention and impact of TCM on diseases and predict the targets and pharmacological effects of TCM, network pharmacology has been proposed and has shown promising results. Network pharmacology, based on the concept of multilevel and multiangle interaction networks of “disease-gene-target-drug,” is consistent with the concept of treating diseases holistically and the principle of a multitarget synergy of TCM and has successfully revealed the pharmacological mechanisms of many TCMs [7].

The active component of JJHYD was first analyzed in this study using UHPLC-MS/MS, and the targets of the active ingredient of JJHYD were screened using network pharmacology. Then, the pharmacological mechanism of the active ingredient of JJHYD was determined using a CHF animal model and cell model.

## 2. Materials and Methods

### 2.1. Composition and Preparation of JJHYD

JJHYD, concocted using *Radix aconiti carmichaeli* (Fuzi) 5 g, dried ginger (Ganjiang) 3 g, *Codonopsis pilosula* (Dangshen) 9 g, *Atractylodes* (Baizhu) 9 g, mature seeds of *Prunus persica (L.) Batsch* (Taoren) 6 g, safflower (Honghua) 6 g, *Glycyrrhizae radix et rhizoma* (Zhigancao) 5 g, were offered by Huamiao Traditional Chinese Medicine Engineering Technology Development Center (Beijing, China). After 30 minutes of immersion in distilled water, the drugs were subjected in an hour of boiling in a 10-fold volume of water. After removing the herbal residue with a filter, the decoctions were obtained.

### 2.2. UHPLC-MS/MS

A 15 mL centrifuge tube was added with JJHYD solution (2 mL) and 10 mL of 50% methanol (*V*/*V*). After 30 minutes of sonication, the supernatant (1 mL) was centrifuged in a clean centrifuge tube at 14,000 rpm for 5 minutes. Then, the resulting supernatant was collected, and subjected to chromatographic separation in a sample vial after being passed through a 0.22 *μ*M microporous membrane. The following were the conditions: mobile phase: A (deionized water, 0.1% formic acid) and B (acetonitrile); chromatographic column: ACQUITY UPLC HSS T3 (2.1 × 100 mm, 1.8 *μ*M, Waters, USA); gradient elution protocol is shown in Supplementary Table 1, flow rate: 0.3 mL/min; injection volume: 10.0 *μ*L; column temperature: 35°C.

Q Exactive Plus Orbitrap high-resolution mass spectrometry (Thermo Fisher, USA) was used for mass spectrometry data acquisition. With Full MS-ddMS^2^ as the detection mode, the negative ion and positive ion modes were scanned using the following conditions: scanning range: m/Z 100-1200, MS^1^ resolution: 70,000, MS^2^ resolution: 17,500, ion source voltage: 3.2 kV, capillary temperature: 320°C, aux gas heater temperature: 350°C, sheath gas flow rate: 40 L/min, aux gas flow rate: 15 L/min, AGC target: 1e6, and topN: 5. The collision energy for triggering the MS2 scan was set to 30, 40, and 50 using a stepped fragmentation voltage NCE.

### 2.3. Identification of Potential Targets of Active Ingredients and HF

Compound discovers 3.2 software was used to extract the characteristic peaks from the RAW mass spectrometric data. The isotope distribution matching, molecular formula prediction, and mass deviation of element matching of the characteristic peaks were all within 5 ppm. For the purpose of identifying characteristic peaks, data from the local self-built mzVault Chinese medicine natural product database and the mzCloud online database (https://www.mzcloud.org/) were utilized. Positive results met the screening criteria of mass deviation <5 ppm, consistent isotope distribution and mzVault best match database matching score > 70. After manual validation and elimination of duplicate results, 227 chemical components were screened. The detected compounds were sequenced by the mass spectral response, and the top 20 compounds were analyzed. The active sources of compounds were retrieved from the Chinese Pharmacopoeia (2015 edition), the literature was inquired from PubMed (https://pubmed.ncbi.nlm.nih.gov/), and the data of compounds were inquired from chemical book, SciFinder database, and PubChem (https://pubchem.ncbi.nlm.nih.gov/). The top 20 compounds are described in Supplementary Table 2.

The potential targets of active ingredients were analyzed by the TCM systems pharmacology database and analysis platform (TCMSP) database (http://sm.nwsuaf.edu.cn/lsp/tcmsp.php) with drug-like properties (DL) ≥ 0.18, oral bioavailability  (OB) ≥ 30%, and the rotatable bonds number (RBN) in the compound <10 as conditions. Zhigancao, which is not included in the TCMSP database, was screened by Bioinformatics Analysis Tool for Molecular mechanism of TCM (BATMAN-TCM) database (http://bionet.ncpsb.org/batman-tcm), and the effective components and targets were determined under the condition that the score cutoff was ≥ 55 and the *q* value was ≤0.05. Therapeutic Target Database (TTD) (http://db.idrblab.net/ttd/) was applied to analyze the potential targets of HF. Twelve potential targets were obtained by intersection.

In order to draw the protein-protein interaction network, the potential action targets were introduced into String (https://www.string-db.org/), using an interaction score > 0.4. The constructed protein-protein interaction network was introduced into Cytoscape 3.7.0, and further analysis of the network was performed by cytoHubba plug-in to obtain key genes. The first 10 key genes were screened based on the MCC algorithm.

### 2.4. Analyses of Gene Ontology (GO) As Well as Kyoto Encyclopedia of Genes and Genomes (KEGG)

GO and KEGG pathway annotations were performed using the GDCRNATools R-package, and the results were visualized.

### 2.5. Molecular Docking

The first five active components with the largest number of targets and the largest number of potential targets were selected as ligands, and their 3D structures were obtained from PubChem. The potential targets they contained (the protein crystal structure of the targets was derived from the PDB database) were molecular docked using the software Autodock Vina, SwissTargetPrediction (http://www.swisstargetprediction.ch/) was applied to predict the ability of active compounds and targets to bind.

### 2.6. Animals and Ethics Statement

Guangdong Medical Laboratory Animal Center (https://www.gdmlac.com.cn/) provided 50 male C57BL/6 mice (8-10 weeks), which were housed in a setting with ambient temperature of 21 ± 0.5°C, humidity of 45-50%, and lighting cycle of light/dark for 12/12 hours. The Experimental Animal Ethics Committee of Shanghai Tenth People's Hospital (SHDSYY-2022-3589) gave its approval to all animal experiments, which were carried out following the guidelines of the China Council on Animal Care and Use.

### 2.7. Groups and Drug Treatment

Five groups of mice, labeled control, Pae-50, CHF, CHF + Pae-20, and CHF + Pae-50, were randomly created. After chronic isoproterenol (ISO, II0200, Solarbio, China, 30 mg/kg/d) infusion for 14 days using osmotic minipumps (2002, Alzet, USA) as previously described [8, 9], the mouse model of CHF was constructed. The mice in the control group and Pae-50 group received intravenous infusions of saline containing 0.002% ascorbic acid for 14 days. After modeling, mice in the Pae-50, CHF + Pae-20, and CHF + Pae-50 groups were intragastrically administered Pae (SP8040, Solarbio, China, 20 or 50 mg/kg/d [10]) every day for a total of 6 days. Normal saline was intragastrically administered to mice in the CHF group every day.

### 2.8. Echocardiography

By inhaling 2% isoflurane, the mice were anesthetized. With the use of VEVO 770 high-resolution imaging system (VisualSonics, Canada), transthoracic echocardiography was carried out. LV end-systolic diameter (LVESD), LV end-diastolic diameter (LVEDD), LV end-diastolic left ventricular posterior wall thickness (LVPWD), interventricular septum diameter (IVSD), LV ejection fraction (LVEF%), and LV fractional shortening (LVFS%) were recorded using two-dimensional M-mode echocardiography.

### 2.9. Cardiac Physiological Index Test Assessment

The tibia length (TL) and body weight (BW) of the mice were measured after euthanasia (pentobarbital solution, 250 mg/kg [11]). The heart of the mice was collected, washed with precooled PBS, and the heart weight (HW) was examined.

### 2.10. Histological Analysis

Fixation of the heart of mice with 10% Neutral buffered Formalin (G2161, Solarbio, China) was conducted, followed by paraffin embedding or frozen sectioning (-15°C). With the help of an H&E kit (BL700A, Biosharp, China), hematoxylin and eosin (H&E) was used for the staining of the paraffin sections, while Oil red O solution (BA4081, BASO, China) for the staining of the frozen sections that were then counterstained with hematoxylin. The sections were observed under a microscope (40× or 200 ×, BX53M, Olympus, Japan), and 5 fields of view were chosen at random from each sample.

### 2.11. Cell Culture and Treatment

Dulbecco's modified eagle medium (DMEM, 11965092, Thermo Fisher, USA) was employed to develop fetal heart cell line CCC-HEH-2 (Type Culture Collection of the Chinese Academy of Sciences, China), which was supplemented with 10% fetal bovine serum (F2442, Sigma-Aldrich, USA) and 1% Penicillin-Streptomycin (P4333, Sigma-Aldrich, USA) with 5% CO_2_ at 37°C.

Glycogen Synthase Kinase-3 alpha (GSK3A) overexpression plasmid (G146459, YouBio, China), empty vector (negative control), PPAR*α* specific small interfering RNA (siPPAR*α*, siB121992833-1-5, Ribobio, China) and siNC (siN0000001-1-5, Ribobio, China) were transfected into CCC-HEH-2 cells with the help of transfection reagent (L3000075, Thermo Fisher, USA). Briefly, CCC-HEH-2 cells were cultured in 6-well plates until 80% confluence. GSK3A overexpression plasmid, siPPAR*α* and transfection reagent were diluted using the Opti-MEM media (31985062, Thermo Fisher, USA) and added to the cells. The medium was changed to DMEM after the cells were cultured for 6 hours. Cells were cultured for 48 hours prior to western blot or qRT-PCR.

Following 30 minutes of pretreatment with Pae (0, 10, 50, 100, 200, and 400 *μ*M [10]), CCC-HEH-2 cells or transfected CCC-HEH-2 cells were incubated with ISO (10 *μ*M [8]) for 24 hours.

### 2.12. qRT-PCR

Using the Total RNA Isolation Reagent (BS259A, Biosharp, China), total RNA was extracted from heart tissues or cells. After that, the total RNA underwent reverse transcription and quantification on a Real-Time PCR system (7500, ThermoFisher, USA) using the One-Step SYBR Green qRT-PCR Kit (BL643B, Biosharp, China). Under the adoption of the 2^−*ΔΔ*CT^ method, B-type natriuretic peptide (BNP), atrial natriuretic peptide (ANP), major histocompatibility complex-B (B-MHC), GSK3A, CD36, PDK4 (Pyruvate dehydrogenase kinase 4), and Cpt1b (carnitine palmitoyltransferase 1B) expressions were normalized to glyceraldehyde-3-phosphate dehydrogenase (GAPDH) [12]. Supplementary Table 3 lists the primer sequences.

### 2.13. Western Blot

Through the use of RIPA lysis buffer (R0010, Solarbio, China), total protein was isolated from tissues and cells, followed by quantification using a BCA protein kit (PC0020, Solarbio, China). In the following step, protein lysates were separated on SDS-PAGE gel prior to being transferred into a polyvinylidene fluoride membrane. Subsequent to 2 hours of blocking, the membrane was added with primary antibodies (4°C, overnight) and secondary antibodies (ambient temperature, 1 hour) for incubation. On the iBright CL750 Imaging System (Thermo Fisher, USA), immunoblots were visualized using an ECL kit (PE0010, Solarbio, China). The antibody information is shown in Supplementary Table 4.

### 2.14. Apoptosis

As for the apoptosis of CCC-HEH-2 cells, an Annexin V-FITC/PI Apoptosis Detection Kit (E606336, Sangon, China) was applied for its evaluation. To be specific, resuspension of CCC-HEH-2 cells at a concentration of 2 × 10^5^ cells/mL in binding buffer was firstly carried out. Then, the cells were mixed in the dark with Annexin V-FITC (5 *μ*L) and PI (10 *μ*L). With the use of a FACSVia flow cytometer (BD, USA), the apoptosis rate was examined.

### 2.15. Statistical Analysis

Mean ± standard deviation was used to express measurement data. Multigroup comparisons were made using one-way analysis of variance (ANOVA). Graphpad 8.0 software was employed for the conduction of statistical analyses, and *P* < 0.05 deemed statistical significant.

## 3. Results

### 3.1. Active Components in JJHYD

The composition of JJHYD was identified by UHPLC-MS/MS. Total ion current (TIC) diagrams are shown in Figures 1(a) and 1(b). Compounds with an mzCloud Best Match Score greater than 70 were screened by comparison with the mzCloud database, and 227 chemical components were obtained after manual validation and elimination of duplicate results. Active information for the top 20 compounds in JJHYD is presented in Supplementary Table 2.

### 3.2. Screening of Target Genes and Construction of a Drug-Ingredient-Target-Disease Network

The TCMSP database yielded a total of 242 target genes for JJHYD, and the TTD database yielded 76 target genes related to HF. Twelve potential action targets were obtained from the intersection of the two databases (Figure 2(a)). We performed network pharmacology analysis on the information obtained on the effective components and targets in JJHYD using Cytoscape 3.7.0 software and established a drug-ingredient-target-disease network (Figure 2(b)). The core nodes were screened according to the sequencing condition of the number of active component targets and the number of active component targets related to HF. The results showed that the core nodes represented the active components including paeonol, apigenin, and luteolin. The first 10 key genes were screened based on the MCC algorithm, and their interaction network is shown in Figure 2(c).

### 3.3. GO and KEGG Enrichment Analyses

The results of GO function analysis showed that JJHYD could exert its anti-HF effects by affecting a variety of biological functions, such as response to drugs, reactive oxygen species metabolism, and oxidative stress. (Figure 3(a)). The KEGG pathway enrichment analysis results revealed the main enrichment of JJHYD in lipids and atherosclerosis, the AGE-RAGE signaling pathway in diabetic complications, fluid shear stress and atherosclerosis, and TNF signaling pathway (Figure 3(b)).

### 3.4. Paeonol Relieved the ISO-Induced Cardiac Dysfunction

The above analysis showed that Pae, apigenin, and mignonette exerted protective effects on the heart, and the content of Pae in JJHYD was the highest. Therefore, we selected Pae for further study. The effects of Pae on the cardiac function of CHF mice were evaluated by echocardiography. ISO-infused mice developed cardiac dysfunction, manifested as increased LVESD, LVEDD, LVPWD, and IVSD as well as decreased LVEF and LVFS (Figures 4(a)–4(f), *P* < 0.001). The cardiac dysfunction of CHF mice was alleviated after treatment with Pae, and CHF mice treated with 50 mg/kg/d Pae showed more efficient remission than CHF mice treated with 20 *μ*M Pae (Figures 4(a)–4(f), *P* < 0.01). However, Pae alone did not affect cardiac function (Figures 4(a)–4(f)).

### 3.5. Paeonol Relieved the ISO-Induced Cardiac Hypertrophy

Relative to the control group, the heart of mice in the CHF group were markedly hypertrophic, manifested as increases in HW/BW and HW/TL, while Pae treatment caused a decline in these two indices (Figures 4(g)–4(h), *P* < 0.01). In addition, the results of H&E staining also indicated the evident cardiac hypertrophy in the CHF Group, but this phenomenon was alleviated by treatment with Pae (Figure 5(a)). Moreover, the increase in markers of myocardial hypertrophy (ANP, BNP, and B-MHC) caused by ISO infusion were reversed by Pae treatment, suggesting that Pae treatment could alleviate ISO-induced cardiac hypertrophy (Figures 5(b)–5(d), *P* < 0.01).

### 3.6. Paeonol Targeted GSK3A and Reduced Cardiac Lipid Accumulation

Molecular docking analysis indicated that Pae might target GSK3A (Figure 5(e)), and SwissTargetPrediction also predicted that Pae could regulate GSK3A. Therefore, we assessed the GSK3A expression in the myocardial tissues in each group. As shown in Figures 5(f)–5(h), Pae treatment reduced the protein levels of GSK3A rather than the mRNA levels of GSK3A (*P* < 0.05). After ISO infusion, the protein and mRNA levels of GSK3A in the myocardial tissue of mice were elevated, while the Pae treatment reduced the protein levels of GSK3A rather than the mRNA levels of GSK3A (Figures 5(f)–5(h), *P* < 0.001). Based on bioinformatics analysis, which revealed that JJHYD was primarily rich in the lipid and atherosclerotic pathways, we determined the effects of Pae on cardiac lipid metabolism, and the results showed that Pae concentration-dependently reduced ISO-induced cardiac lipid accumulation (Figure 5(j)).

### 3.7. Overexpression of GSK3A Reversed the Inhibitory Effect of Paeonol on Cardiac Lipid Accumulation *In Vitro*

The human cardiomyocytes CCC-HEH-2 were used to construct CHF cell models to verify the effects of Pae on CHF. Pae dose-dependently inhibited the protein levels of GSK3A in CCC-HEH-2 cells (Figures 6(a) and 6(b), *P* < 0.01), so concentrations of 100 *μ*M and 400 *μ*M were chosen for the following experiments. CCC-HEH-2 cells treated with ISO not only expressed more GSK3A (Figures 6(c) and 6(d), *P* < 0.001) but also showed more lipid accumulation than the control group (Figures 6(e) and 6(f), *P* < 0.001). However, Pae pretreatment significantly alleviated these conditions, with the effect of 400 *μ*M Pae being more significant (Figures 6(c)–6(f), *P* < 0.05). Interestingly, the inhibitory effects of Pae pretreatment on GSK3A protein and lipid accumulation were reversed by GSK3A overexpression (Figures 6(g)–6(j), *P* < 0.001), which indicated that Pae reduced the lipid accumulation of cardiomyocytes by reducing the protein levels of GSK3A.

### 3.8. Overexpression of GSK3A Reversed the Inhibitory Effects of Paeonol on the Activation of the PPAR*α* Signaling Pathway *In Vitro*

Since PPAR*α* transcription factors play a major role in regulating cardiac fatty acid metabolism, we detected PPAR*α* and its downstream target gene expressions. After ISO treatment of CCC-HEH-2 cells, the expression levels of p-PPAR*α*, PPAR*α*, p-PPAR*α*/PPAR*α* (Figures 7(a)–7(d)), and PPAR*α* downstream genes (CD36, Cpt1b, and PDK4) (Figure 7(i)) were significantly increased (*P* < 0.001), but this trend was reversed with Pae treatment (*P* < 0.001). However, the reversal effect of Pae was offset by GSK3A overexpression (Figures 7(e)–7(h) and 7(j), *P* < 0.001).

### 3.9. SiPPAR*α* Reversed the Effects of GSK3A Overexpression on CCC-HEH-2 Cells *In Vitro*

To determine whether GSK3A promoted myocardial lipid deposition by activating the PPAR*α* pathway, we used siPPAR*α* to silence PPAR*α*. GSK3A overexpression plasmid facilitated the expression levels of p-PPAR*α*, PPAR*α*, p-PPAR*α*/PPAR*α*, and PPAR*α* downstream genes (CD36, Cpt1b, and PDK4), while siPPAR*α* did the opposite (Figures 8(a)–8(e), *P* < 0.001). The cotransfection of GSK3A overexpression plasmid and siPPAR*α* neutralized the effects of GSK3A overexpression or siPPAR*α* on PPAR*α* pathway-related proteins or genes (Figures 8(a)–8(e), *P* < 0.05). In addition, ISO-induced lipid deposition (Figures 8(f) and 8(g)) and apoptosis (Figures 8(h) and 8(i)) in cardiomyocytes were enhanced by GSK3A overexpression and inhibited by siPPAR*α* (*P* < 0.01). Similarly, both the effects of GSK3A overexpression and the effects of siPPAR*α* were reversed by cotransfection of the two (Figures 8(f)–8(i), *P* < 0.01).

## 4. Discussion

TCM theory states that CHF is included in the syndrome of blood stasis and qi deficiency [4]. JJHYD, a blend of seven herbal medicines, effectively treats the signs and symptoms of CHF while lowering toxicity. In this study, we used UHPLC-MS/MS analysis along with database retrieval to pinpoint the primary active ingredients of JJHYD. One of these active ingredients, hydroxysafflor yellow A, demonstrated effects that encouraged blood circulation to remove blood stasis [13], baicalin, liquiritin, and diammonium glycyrrhizinate demonstrated anti-inflammation and immune regulation effects [14, 15], and paeoniflorin showed antioxidation effects [16]. These results provide a pharmacological basis for JJHYD in treating cardiac diseases. Through network pharmacology analysis, we confirmed that paeonol, apigenin, and luteolin, which have cardioprotective effects, are the potential active ingredients of JJHYD for treating CHF. Among them, the content of paeonol in JJHYD was the highest. Existing literature reveals that paeonol exerts its anti-inflammatory effects by promoting vasodilation and antioxidation and affects the electrophysiological properties of ventricular myocytes [12, 17, 18]; however, it remained undetermined whether these effects could prevent and treat CHF.

We found that JJHYD is mainly enriched in lipids and atherosclerotic pathways through GO and KEGG analyses. Disorders of lipid metabolism are crucial in the etiology of CHF. Under normal circumstances, free fatty acids provide 70% of the energy of cardiomyocytes, while under pathological conditions, the utilization of fatty acids decreases, the synthesis of triglycerides and cholesterol increases, and lipids accumulate in the heart, which causes cardiac hypertrophy and induces the permeability of the mitochondrial membrane to increase, resulting in cardiomyocyte apoptosis [19]. In this study, we established a CHF animal model by infusing ISO into mice. ISO is a *β*-adrenergic receptor agonist. Continuous infusion of ISO increased the heart rate, hemodynamic pressure and contractility, resulting in cardiac hypertrophy and myocardial damage, which is very similar to the pathological changes of CHF [20, 21]. Consistent with previous studies, in our study, ISO induced cardiac dysfunction, cardiac hypertrophy, increased the release of B-MHC, BNP, and ANP, and caused excessive accumulation of cardiac lipids in CHF mice. However, these pathological changes induced by ISO were reversed by paeonol. A similar conclusion has been shown by Li et al., who combined paeonol and danshensu to improve ISO-induced cardiac hypertrophy, cardiac dysfunction, and cardiomyocyte apoptosis [22].

One of the important achievements of this study was identifying the target GSK3A of paeonol through molecular docking and *in vitro* experiments. GSK3A, an isoform of serine/threonine kinase GSK3, is highly conservative in mammals and involved in cell apoptosis and mitosis [23]. Importantly, GSK3A contributes significantly to both heart development and heart disease [24]. It was found that the absence of GSK3A restricted cardiac dysfunction and cardiomyocyte apoptosis, promoted cardiomyocyte proliferation, and alleviated atherosclerosis [25]. In addition, GSK3A can also regulate the accumulation of fatty acids in the heart. On the one hand, fatty acid accumulation induces the upregulation of GSK3A, while on the other hand, an increase in GSK3A can enhance the absorption and accumulation of fatty acids in the heart [26]. Consistent with the previous findings, we found that the inhibitory effects of paeonol on cardiac lipid accumulation were reversed by GSK3A, suggesting that paeonol resisted cardiolipid toxicity by inhibiting the expression of GSK3A.

Although the exact mechanism via which paenol exerts its effects remains unknown, several mechanisms were proposed in previous literature. When paeonol was tested for its effects and underlying processes on HF brought on by transverse aortic constriction (TAC) in mice, Chen et al. discovered that paeonol attenuated TAC-induced HF via ERK1/2 signaling [27]. In another study using doxorubicin-induced CHF-modeled rats, Chen et al. investigated whether miR-21-5p participated in treating CHF through paeonol [28]. They reported that paeonol exerted cardioprotective effects on CHF caused by doxorubicin via controlling the miR-21-5p/SKP2 axis. Comparatively, we focused on the PPAR*α* pathway associated with cardiac fatty acid metabolism. The PPAR*α* expression level is relatively high in the heart, which regulates the expression of most genes encoding fatty acid transport and oxidation in heart mitochondria at the transcription level, such as CD36, Cpt1b, and PDK4, so activating PPAR*α* can enhance the intracellular fatty acid oxidation process [29]. Notably, GSK3A promoted the accumulation of heart fatty acids through PPAR*α*. Nakamura et al. used heart-specific GSK3A knockdown mice and mutant PPAR*α* mice to prove the promotion of GSK3A/PPAR*α* in lipotoxic cardiomyopathy [26]. In addition to inducing fatty acid accumulation, GSK3A/PPAR*α* can also open the mitochondrial permeability transition pole by recruiting Bax, thus aggravating HF [30, 31]. In our study, the promotion of lipid accumulation and apoptosis by overexpression of GSK3A was reversed by siPPAR*α*, further proving fresh information on the critical function of GSK3A/PPAR*α* in cardiac toxicity.

## 5. Conclusions

In summary, this study illustrates the pharmacological mechanism of paeonol, the main active ingredient of JJHYD, on treating CHF, which specifically targets GSK3A to inhibit the PPAR*α* pathway to prevent cardiac lipid accumulation. This mechanism provides a rationale for developing corresponding inhibitors as a novel therapeutic strategy to improve the outcomes of CHF treatment.

## Figures and Tables

**Figure 1:** TIC diagram of sample extract of JJHYD using ultrahigh-performance liquid chromatography-mass spectrometry in (a) positive ion mode and (b) negative ion mode. TIC: total ion chromatography.

**Figure 2:** Potential target genes of JJHYD and heart failure. (a) Twelve genes were obtained from the intersection of 242 possible targets of JJHYD revealed in the TCMSP database (http://sm.nwsuaf.edu.cn/lsp/tcmsp.php), of which 76 genes were found associated with heart failure from the TTD (http://db.idrblab.net/ttd/). (b) The network of ingredient-target-disease relation. Drugs are represented by the yellow nodes, active ingredients by the blue nodes, diseases by the red nodes, and drug and disease targets by the green nodes. (c) The interaction network of the identified target. JJHYD: Jijiuhuiyang decoction; TCMSP: the traditional Chinese medicine systems pharmacology database and analysis platform; TTD: therapeutic target database.

**Figure 3:** Results of GO and KEGG enrichment analyses. (a) GO enrichment analysis of JJHYD targets in treating CHF. (b) KEGG enrichment analysis of the possible pathways associated with JJHYD in treating CHF. GO: Gene Ontology; KEGG: Kyoto Encyclopedia of Genes and Genomes; CHF: chronic heart failure; JJHYD: Jijiuhuiyang decoction.

**Figure 4:** The effects of paeonol on the heart function of ISO-induced CHF mice. The (a) LVESD, (b) LVEDD, (c) LVPWD, (d) IVSD, (e) LVEF, and (f) LVFS were measured based on long-axis M-mode echocardiography. (g) The heart-to-body weight ratio of the mouse. (h) The ratio of the weight of the mouse's heart to the length of the tibia. ^∗∗∗^*P* < 0.001*vs*. Pae-50 group. ^##^*P* < 0.01, ^###^*P* < 0.001*vs*. CHF group. Pae: paeonol; ISO: isoproterenol; CHF: chronic heart failure; LVESD: left ventricular end-systolic diameter; LVEDD: left ventricular end-diastolic diameter; LVPWD: end-diastolic left ventricular posterior wall thickness; IVSD: interventricular septal thickness in diastole. LV fractional shortening (LVFS%) and LV ejection fraction (LVEF%) were recorded by two-dimensional M-mode echocardiography. TL: tibia length; BW: body weight; HW: heart weight.

**Figure 5:** Paeonol downregulated GSK3A and relieved myocardial hypertrophy and cardiac lipid accumulation in CHF mice. (a) Representative hematoxylin-eosin staining of mouse hearts from the five groups (magnification, 40×, scale bar = 600 *μ*M). The mRNA levels of (b) ANP, (c) BNP, and (d) B-MHC (markers of myocardial hypertrophy) determined by qRT-PCR, taking GAPDH as the internal control. (e) Macromolecular docking diagram of Pae and GSK3A. (f) The protein levels of GSK3A and (g) corresponding quantitative bar chart determined by western blot. (h) The mRNA levels of GSK3A determined by qRT-PCR, taking GAPDH as the internal control. (i) Representative Oil red O staining of cardiac lipid accumulation from the five groups and (j) corresponding histological slides (magnification, 200×, scale bar = 50 *μ*M). ^^^*P* < 0.05*vs*. control group. ^∗∗∗^*P* < 0.001*vs*. Pae-50 group. ^###^*P* < 0.001*vs*. CHF group. Pae: paeonol; CHF: chronic heart failure; GSK3A: Glycogen Synthase Kinase-3 alpha; ANP: atrial natriuretic peptide; BNP: B-type natriuretic peptide; B-MHC: major histocompatibility complex-B; GAPDH: glyceraldehyde-3-phosphate dehydrogenase.

**Figure 6:** Overexpression of GSK3A reversed the inhibitory effect of paeonol on ISO-induced lipid accumulation in human cardiomyocytes. CCC-HEH-2 cells receiving different concentrations of Pae for 30 minutes, (a) the GSK3A protein expression detected by western blot and (b) their corresponding quantitative bar chart, taking GAPDH as the internal control. (c, d) CCC-HEH-2 cells pretreated with or without Pae (100, 400 *μ*M) for 30 minutes and then subjected to a 24 hours of incubation with ISO (10 *μ*M), and the GSK3A expression level assessed by western blot. (e, f) The lipid accumulation detected by Oil red O staining (magnification, 200×, scale bar = 50 *μM*). (g, h) CCC-HEH-2 cells transfected with GSK3A overexpression plasmid or NC pretreated with or without Pae (400 *μ*M) for 30 minutes and then subjected to a 24 hours of incubation with ISO (10 *μ*M), and the GSK3A expression level determined by western blot, (i, j) the lipid accumulation examined by Oil red O staining (magnification, 200×, scale bar = 50 *μ*M). ^∗∗^*P* < 0.01, ^∗∗∗^*P* < 0.001*vs*. blank group. ^#^*P* < 0.05, ^###^*P* < 0.001*vs*. ISO group. ^&&&^*P* < 0.001*vs*. ISO + Pae-400 group. Pae: paeonol; GSK3A: Glycogen Synthase Kinase-3 alpha; ISO: isoproterenol; GAPDH: glyceraldehyde-3-phosphate dehydrogenase; NC: negative control.

**Figure 7:** Overexpression of GSK3A reversed paeonol's inhibitory effect on ISO-induced PPAR*α* pathway activation. (a–d) CCC-HEH-2 cells pretreated with or without Pae (100, 400 *μ*M) for 30 minutes and then subjected to a 24 hours of incubation with ISO (10 *μ*M), and the p-PPAR*α* (b), PPAR*α* (c) and the ratio of p-PPAR*α*/PPAR*α* (d) protein levels measured by western blot. (e–h) Taking GAPDH as the internal control, CCC-HEH-2 cells transfected with GSK3A overexpression plasmid or NC pretreated with or without Pae (400 *μ*M) for 30 minutes and then subjected to a 24 hours of incubation with ISO (10 *μ*M), and the p-PPAR*α*, PPAR*α*, and the ratio of p-PPAR*α*/PPAR*α* protein levels determined by western blot. (i) the mRNA levels of CD36, Cpt1b, and PDK4 (PPAR*α* downstream target genes) obtained by qRT-PCR. (j) the mRNA levels of CD36, Cpt1b, and PDK4 (PPAR*α* downstream target genes) determined by qRT-PCR, with GAPDH being the internal control. ^∗∗∗^*P* < 0.001*vs*. blank group. ^###^*P* < 0.001*vs*. ISO group. ^&&&^*P* < 0.001*vs*. ISO + Pae-400 group. Pae: paeonol; GSK3A: Glycogen Synthase Kinase-3 alpha; ISO: isoproterenol; GAPDH: glyceraldehyde-3-phosphate dehydrogenase; NC: negative control; Cpt1b: carnitine palmitoyltransferase 1B; PDK4: pyruvate dehydrogenase kinase 4.

**Figure 8:** SiPPAR*α* reversed the regulation of GSK3A overexpression on the PPAR*α* pathway activation, lipid accumulation, and apoptosis. (a–d) CCC-HEH-2 cells transfected with NC or GSK3A overexpression plasmid or cotransfected with GSK3A overexpression plasmid/NC and siPPAR*α*, the p-PPAR*α* and PPAR*α* protein levels as well as the ratio of p-PPAR*α*/PPAR*α* measured by western blot. (e) The mRNA levels of CD36, Cpt1b, and PDK4 (PPAR*α* downstream target genes) assessed by qRT-PCR. (f, g) The lipid accumulation detected by Oil red O staining (magnification, 200×, scale bar = 50 *μ*M). (h, i) The apoptosis rate determined by flow cytometry. ^∗∗∗^*P* < 0.001*vs*. NC group. ^##^*P* < 0.01, ^###^*P* < 0.001*vs*. GSK3A group. ^^^*P* < 0.05, ^^^^*P* < 0.01, ^^^^^*P* < 0.001*vs*. NC+ siPPAR*α* group. Pae: paeonol; GSK3A: Glycogen Synthase Kinase-3 alpha; ISO: isoproterenol; GAPDH: glyceraldehyde-3-phosphate dehydrogenase; NC: negative control.

## Data Availability

The analyzed data sets generated during the study are available from the corresponding author on reasonable request.

## Additional Points

*Highlights*. (1) Paeonol was identified as the highest content ingredient among JJHYD's heart-protecting active ingredients. (2) Paeonol alleviated ISO-induced cardiac dysfunction, cardiac hypertrophy, and myocardial lipid accumulation. (3) Paeonol inhibited the activation of the PPAR*α* pathway by targeting GSK3A.

## Supplementary Materials

Supplementary materials Supplementary Table 1: gradient elution protocol. Supplementary Table 2: effective chemical constituents and targets of JiJiu Huiyang decoction (top 20). Supplementary Table 3: primers used in this study. Supplementary Table 4: antibodies used for western blot.

## References

[1] Skrzypek A., Mostowik M., Szeliga M., Wilczynska-Golonka M., Debicka-Dabrowska D., Nessler J. (2018). Chronic heart failure in the elderly: still a current medical problem. *Folia Medica Cracoviensia*.

[2] Yao Y. S., Li T. D., Zeng Z. H. (2020). Mechanisms underlying direct actions of hyperlipidemia on myocardium: an updated review. *Lipids in Health and Disease*.

[3] Mazurek J. A., Jessup M. (2015). Understanding heart failure. *Cardiac Electrophysiology Clinics*.

[4] Wang Y., Wang Q., Li C. (2017). A review of Chinese herbal medicine for the treatment of chronic heart failure. *Current Pharmaceutical Design*.

[5] Gai Q. Y., Jiao J., Wang X. (2020). Simultaneous determination of taxoids and flavonoids in twigs and leaves of three _Taxus_ species by UHPLC-MS/MS. *Journal of Pharmaceutical and Biomedical Analysis*.

[6] Xu Y., Yang L., Liang K., An R., Wang X., Zhang H. (2020). Pharmacokinetic effects of ginsenoside Rg1 on aconitine, benzoylaconine and aconine by UHPLC-MS/MS. *Biomedical Chromatography*.

[7] Hu Q., Wei S., Wen J. (2020). Network pharmacology reveals the multiple mechanisms of Xiaochaihu decoction in the treatment of non-alcoholic fatty liver disease. *BioData Mining*.

[8] Yang Y., Xu C., Tang S., Xia Z. (2020). Interleukin-9 aggravates isoproterenol-induced heart failure by activating signal transducer and activator of transcription 3 signalling. *The Canadian Journal of Cardiology*.

[9] Zhou Q., Pan L. L., Xue R. (2020). The anti-microbial peptide LL-37/CRAMP levels are associated with acute heart failure and can attenuate cardiac dysfunction in multiple preclinical models of heart failure. *Theranostics*.

[10] Wu J., Sun C., Wang R. (2018). Cardioprotective effect of paeonol against epirubicin-induced heart injury via regulating miR-1 and PI3K/AKT pathway. *Chemico-Biological Interactions*.

[11] Dutton J. W., Artwohl J. E., Huang X., Fortman J. D. (2019). Assessment of pain associated with the injection of sodium pentobarbital in laboratory mice (Mus musculus). *Journal of the American Association for Laboratory Animal Science*.

[12] Zheng J., Mao Z., Zhang J., Jiang L., Wang N. (2020). Paeonol pretreatment attenuates anoxia-reoxygenation induced injury in cardiac myocytes <i>via</i> a BRCA1 dependent pathway. *Chemical and Pharmaceutical Bulletin (Tokyo)*.

[13] Bai X., Wang W. X., Fu R. J. (2020). Therapeutic potential of Hydroxysafflor yellow a on cardio-cerebrovascular diseases. *Frontiers in Pharmacology*.

[14] Xin L., Gao J., Lin H. (2020). Regulatory mechanisms of baicalin in cardiovascular diseases: a review. *Frontiers in Pharmacology*.

[15] Sharifi-Rad J., Quispe C., Herrera-Bravo J. (2021). Glycyrrhiza genus: enlightening phytochemical components for pharmacological and health-promoting abilities. *Oxidative Medicine and Cellular Longevity*.

[16] Zhang Y., Wu X., Wang X. (2021). Grey relational analysis combined with network pharmacology to identify antioxidant components and uncover its mechanism from Moutan Cortex. *Frontiers in Pharmacology*.

[17] Ma L., Chuang C. C., Weng W. (2016). Paeonol protects rat heart by improving regional blood perfusion during no-reflow. *Frontiers in Physiology*.

[18] Ma Y. L., Bates S., Gurney A. M. (2006). The effects of paeonol on the electrophysiological properties of cardiac ventricular myocytes. *European Journal of Pharmacology*.

[19] Azevedo P. S., Minicucci M. F., Santos P. P., Paiva S. A., Zornoff L. A. (2013). Energy metabolism in cardiac remodeling and heart failure. *Cardiology in Review*.

[20] Branco A. F., Moreira A. C., Cunha-Oliveira T. (2014). *β*-Adrenergic over-stimulation and cardio-myocyte apoptosis: two receptors, one organelle, two fates?. *Current Drug Targets*.

[21] Cheng H., Wu X., Ni G. (2020). Citri Reticulatae Pericarpium protects against isoproterenol-induced chronic heart failure via activation of PPAR*γ*. *Annals of Translational Medicine*.

[22] Li H., Xie Y. H., Yang Q. (2012). Cardioprotective effect of paeonol and danshensu combination on isoproterenol-induced myocardial injury in rats. *PLoS One*.

[23] Kaidanovich-Beilin O., Woodgett J. R. (2011). GSK-3: functional insights from cell biology and animal models. *Frontiers in Molecular Neuroscience*.

[24] Takahashi-Yanaga F. (2018). Roles of glycogen synthase kinase-3 (GSK-3) in cardiac development and heart disease. *Journal of UOEH*.

[25] Ahmad F., Woodgett J. R. (2020). Emerging roles of GSK-3*α* in pathophysiology: emphasis on cardio-metabolic disorders. *Biochimica et Biophysica Acta: Molecular Cell Research*.

[26] Nakamura M., Liu T., Husain S. (2019). Glycogen synthase kinase-3alpha promotes fatty acid uptake and lipotoxic cardiomyopathy. *Cell Metabolism*.

[27] Chen X., Zhang Z., Zhang X. (2022). Paeonol attenuates heart failure induced by transverse aortic constriction via ERK1/2 signalling. *Pharmaceutical Biology*.

[28] Chen C., Liu S., Cao G. (2022). Cardioprotective effect of paeonol on chronic heart failure induced by doxorubicin via regulating the miR-21-5p/S-phase kinase-associated protein 2 axis. *Frontiers in Cardiovascular Medicine*.

[29] Han L., Shen W. J., Bittner S., Kraemer F. B., Azhar S. (2017). PPARs: regulators of metabolism and as therapeutic targets in cardiovascular disease. Part II: PPAR-*β*/*δ* and PPAR-*γ*. *Future Cardiology*.

[30] Ahmad F., Singh A. P., Tomar D. (2019). Cardiomyocyte-GSK-3*α* promotes mPTP opening and heart failure in mice with chronic pressure overload. *Journal of Molecular and Cellular Cardiology*.

[31] Kwong J. Q., Molkentin J. D. (2015). Physiological and pathological roles of the mitochondrial permeability transition pore in the heart. *Cell Metabolism*.

